# Feature Selection on Elite Hybrid Binary Cuckoo Search in Binary Label Classification

**DOI:** 10.1155/2021/5588385

**Published:** 2021-05-11

**Authors:** Maoxian Zhao, Yue Qin

**Affiliations:** College of Mathematics and Systems Science, Shandong University of Science and Technology, Qingdao, Shandong 266590, China

## Abstract

For the low optimization accuracy of the cuckoo search algorithm, a new search algorithm, the Elite Hybrid Binary Cuckoo Search (EHBCS) algorithm, is improved by feature weighting and elite strategy. The EHBCS algorithm has been designed for feature selection on a series of binary classification datasets, including low-dimensional and high-dimensional samples by SVM classifier. The experimental results show that the EHBCS algorithm achieves better classification performances compared with binary genetic algorithm and binary particle swarm optimization algorithm. Besides, we explain its superiority in terms of standard deviation, sensitivity, specificity, precision, and *F*-measure.

## 1. Introduction

Feature selection attempts to find the most discriminative subset of features to bring reasonable recognition rates for some classifiers. Given a problem with *d* features, we have 2^*d*^ possible solutions, making an exhaustive search impracticable for high-dimensional feature spaces. In addition, the high-dimensional data also contains a large number of irrelevant and noise-polluted features, and there is often information redundancy between features. These factors will affect the learning effect of the learning algorithm and significantly increase the algorithm's computational complexity. Therefore, feature selection has become a research hot spot.

As a key technology of pattern recognition and machine learning, feature selection is an effective method to deal with high-dimensional data. Feature selection models can be divided into three categories [1]: filter [2], embedding [3], and wrapper [4]. Filter methods define the relevant features without prior classification of the data. The embedding method refers to the process of embedding the feature selection algorithm into the classification algorithm and conducting feature selection and training at the same time. Wrapper methods on the other hand incorporate classification algorithms to search for and select relevant features. The wrapper methods generally outperform filter methods in terms of classification accuracy [5]. Recent studies have shown that feature selection can better solve many practical problems, including classification and medical problems [6–9].

Another vital part of the feature selection process is the search strategy: selecting the feature subset that meets the optimal evaluation criteria, which is usually a combinatorial optimization problem. In recent years, metaheuristic algorithms based on biological behavior and physical systems in nature are proposed to solve the optimization problems [10]. Metaheuristic optimization algorithm, also known as natural heuristic algorithm, studies the evolutionary behavior of species and simulates it into computer science algorithms, including genetic algorithm [11], particle swarm optimization algorithm [12], bat algorithm [13, 14], and cuckoo algorithm [15]. The metaheuristic optimization algorithm has achieved good results in feature selection. For example, Liu et al. [16] combined genetic algorithm and simulated annealing algorithm to select feature subsets. The experiment result expresses the hybrid algorithm has high reliability and strong convergence. On the contrary, Siedlecki and Sklansky [17] combined genetic algorithm and feature selection to achieve a certain effect, but it exposed the problem of premature convergence of genetic algorithm. Kennedy and Eberhart [18] proposed the binary particle swarm optimization algorithm called BPSO, which modified the traditional particle swarm optimization algorithm and solves the binary optimization problems. Besides, Firpi and Goodman [19] applied BPSO to feature selection problems.

The success of metaheuristic methods lies in the efficiency of search strategies and its ability to find solutions to combinatorial optimization problems. Metaheuristics take the information gathered during the search to guide the search process, and therefore, they are considered independent of the problems. The cuckoo search algorithm is a novel heuristic optimization approach introduced by Yang and Deb in 2009 [15]. The algorithm simulates cuckoo birds' parasitic breeding habits and is a random algorithm with strong global search ability. The cuckoo search algorithm has been efficiently employed in many fields, such as intelligent optimization and calculation. Cuckoo search is superior to other algorithms in continuous optimization problems including spring design and welding beam in engineering design applications [20]. This algorithm is especially suitable for large-scale problems [21]. Valian et al. have applied it in training the neural network [22] and spike neural model [23]. The experiment proved that CS has better search capability than other algorithms like particle swarm optimization algorithm, genetic algorithm, and artificial bee colony algorithm [21, 24, 25]. Therefore, CS is a metaheuristic algorithm used in combinatorial optimization problems to obtain higher performance.

The CS can only solve optimization problems in the continuous solution space. To solve combinatorial optimization problems in discrete solution space, Gherboudj et al. [26] proposed a binary version of the cuckoo search algorithm, namely, BCS algorithm. Pereira and Rodrigues [27] applied BCS algorithm to feature selection. Bhattacharjee and Sarmah [28] improved BCS by using the balance combination of local random walk and global exploration random walk so that BCS algorithm can better balance locality and globality. Sudha and Selvarajan [29] presented a feature selection approach based on an enhanced cuckoo algorithm and applied it to breast X-ray images. It can supply valuable information for clinicopathologists. Aziz and Hassanien [30] proposed a new improved cuckoo algorithm combined with the theoretical knowledge of rough set and finally applied it to feature selection.

The cuckoo search algorithm uses Lévy flight random walk to search space in the iteration. The cuckoo search cannot effectively search around the cuckoo's nest due to the Lévy flight with sharp 90-degree turns. Therefore, it suffers from low optimization accuracy [31]. In order to improve the cuckoo search algorithm, this paper proposes an Elite Hybrid Binary Cuckoo Search algorithm, and the novelty of the paper is two-fold:

1. EHBCS adopts feature weighting and elite strategy in the binary cuckoo search algorithm. Feature weighting based on Relief algorithm is to estimate the feature weight and its importance according to the ability of each feature to distinguish different class instances. Elite strategy and genetic algorithm with the selection and crossover operators are embedded into the cuckoo algorithm so that the well-positioned nests can be inherited to the next generation
2. EHBCS is applied to a set of binary label datasets, including low-dimensional and high-dimensional samples such that only the best features are retained in the subset. Experimental results demonstrate that EHBCS achieves a better classification performance to minimize the number of selected features, simultaneously maximizing the classification accuracy by SVM compared with binary genetic algorithm and binary particle swarm optimization

The main contributions of this paper are summarized as follows: (1) It is the first time to combine the feature weighting and elite strategy with BCS algorithm. (2) It specifically improves the low optimization accuracy of the BCS algorithm. (3) It may provide a useful revelation to high-dimensional data researches such as text processing, medical research, and gene analysis.

The structure of this paper is as follows: Section 2 provides details of the classical version of the Cuckoo Search and Binary Cuckoo Search algorithms; Section 3 presents the Elite Hybrid Binary Cuckoo Search (EHBCS) algorithm; Section 4 discusses the experimental methodology and in particular the dataset and evaluation measures; numerical experiment is also carried out to evaluate the prediction performance of our method in Section 5. The results demonstrate that the proposed method is efficient for high-dimensional datasets; finally, the conclusions of our work are given in Section 6.

## 2. Cuckoo Search Algorithm

### 2.1. Cuckoo Search (CS) Algorithm

The parasite behavior of cuckoos is extremely intriguing. These birds can lay down their eggs in host nests and mimic external characteristics of host eggs such as color and spots. If this strategy is unsuccessful, the host can throw the cuckoo's eggs away or simply abandon its nest, making a new one in another place. Based on this context, Yang and Deb [15] have developed a novel evolutionary optimization algorithm named cuckoo search (CS), and they have summarized CS using three rules, as follows:

1. Each cuckoo chooses a nest to lays eggs randomly
2. The number of available host nests is fixed, and nests with high-quality eggs will be passed on the next generations
3. If a host bird discovered the cuckoo egg, it can throw the egg away or abandon the nest and build a completely new nest

For optimization problems, each nest represents a possible solution to the problems, and a nest can contain one or more eggs depending on the size of the problems. Firstly, the algorithm randomly initializes each nest, and then, the algorithm carries out an iterative process. During each iteration, each nest is updated by Lévy flight with random walk, and the formula is shown in Equations (1) and (2):

(1) $$\begin{array}{c} x_{i}^{t+1}=x_{i}^{t}+\alpha ⊕{\text{le}}^{\prime }\text{vy}\left(\lambda \right). \end{array}$$

The updating formula of each dimension is expressed as

(2) $$\begin{array}{c} x_{ij}^{t+1}=x_{ij}^{t}+\alpha \times {\text{le}}^{\prime }\text{v}{\text{y}}_{j}\left(\lambda \right), \end{array}$$

where *x*_*i*_^*t*^ denotes *i*th nest and *x*_*ij*_^*t*^ stands for the *j*th eggs at nest *i* for the *t* generation. *α* is step size, and the product ⊕ means entrywise multiplications. In most case, we can use *α* = 1. The Lévy flights Lévy (*λ*) employ a random step length, and Lévy _*j*_(*λ*) is its *j*th component.

In the 1930s, Lévy proposed Lévy's distribution, believing that the relationship between the continuous jump path of Lévy's flight and time *t* follows Lévy's distribution. Later, many scholars have studied Lévy's distribution and used it to explain random phenomena in nature, such as Brownian motion and random walk. Yang [15] studied and obtained the probability density function of Lévy distribution in power form by simplifying and Fourier transform:

(3) $$\begin{array}{c} {\text{le}}^{\prime }\text{vy}\sim u=t^{-\lambda }\left(1<\lambda \leq 3\right), \end{array}$$

where *λ* is the power coefficient. Equation (2) is a probability distribution with a heavy tail. Although it can essentially describe the random walk process of cuckoo birds, it has not been further described in a more concise and easy to program mathematical language to achieve the CS algorithm. So Yang adopted the Mantegna algorithm to simulate Lévy jump path:

(4) $$\begin{array}{c} s=\frac{u}{{\left|v\right|}^{1/\beta }}, \end{array}$$

where *s* is the Lévy flight Lévy _*j*_(*λ*), the relation of parameters *β* in equation (2) is *λ* = 1 + *β* and content 0<*β*≤2. The parameter is *β* = 1.5, and *μ* and *ν* are random number and satisfy Equations (5) and (6):

(5) $$\begin{array}{c} \left\{\begin{array}{c} \mu \sim N\left(0,\sigma_{\mu }^{2}\right)\\ \nu \sim N\left(0,\sigma_{\nu }^{2}\right) \end{array},\right. \end{array}$$

(6) $$\begin{array}{c} \left\{\begin{array}{c} \begin{array}{c} \sigma_{\mu }={\left\{\frac{\Gamma \left(1+\beta \right)\cdot \sin\left(\beta \pi /2\right)}{\Gamma \left(1+\beta /2\right)\cdot \beta \cdot 2^{\left(\beta -1\right)/2}}\right\}}^{1/\beta },\\ \sigma_{\nu }=1. \end{array} \end{array}\right. \end{array}$$

Let $\text{step}=\alpha \times \text{l}\overset{´}{\text{e}}\text{vy}{\left(\lambda \right)}_{j}=\alpha \times s$ then step is the path that cuckoo bird experiences each time in solution space when it randomly searches for the new nest location *x*_*ij*_^*t*+1^ from the old nest location *x*_*ij*_^*t*^ according to Equation (2). In the finally step of each iteration, the nest with the worst quality is substituted with probability p _*a*_∈[0,1].  Algorithm 1 shows the pseudo-code for the classical version of CS.

### 2.2. Binary Cuckoo Search (BCS) Algorithm

In traditional CS, the position of the solution is updated in the continuous search space. Unlike the above CS, the BCS search space for feature selection is modeled as a binary *d*-bit string, where *d* is the number of features. BCS represents each nest as a binary vector, where each 1 corresponds to a selected feature and 0 otherwise. This means each nest represents a possible solution, and each nest represents a feature.

(7) $$\begin{array}{c} x_{ij}=\left\{\begin{array}{cc} 1 & x_{i}\text{ selects the }j\text{th feature}\\ 0 & \text{otherwise} \end{array}.\right. \end{array}$$

The original cuckoo algorithm introduces mapping functions to extend the cuckoo algorithm to discrete binary regions as follows [25]:

(8) $$\begin{array}{c} \text{sig}\left(\text{step}\right)=\frac{1}{1+e^{-\gamma \text{step}}},\gamma =1, \end{array}$$

(9) $$\begin{array}{c} x_{ij}^{t}=\left\{\begin{array}{c} \begin{array}{cc} 1 & \mathrm{rand}\left(\right)\leq \text{sig}\left(\text{step}\right)\\ 0 & \text{otherwise} \end{array}, \end{array}\right. \end{array}$$

in which rand() ~ *U*(0, 1) and *x*_*ij*_^*t*^ denotes the new egg's value at iteration *t*.

## 3. Elite Hybrid Binary Cuckoo Search (EHBCS) Algorithm

### 3.1. Feature Weighting Based on Relief Algorithm

The core idea of feature weighting based on Relief is to estimate the feature weight and its importance according to the ability of each feature to distinguish different class instances [32]. Given a two-class dataset *D*, *C* containing *n* cases is a class label set, *x* = (*x*_1_, *x*_2_, ⋯, *x*_*d*_) is a case in *D*, and *x* is a real-valued vector with dimension *d*. Relief performs the following iterative learning: randomly select a case *x*, then find the nearest case NH(*x*) of the same class and the nearest case NM(*x*) of the different class, and then update the weight using the following rules:

(10) $$\begin{array}{c} w_{j}=w_{j}+\frac{1}{T}\left|x_{j}-\text{NM}{\left(x\right)}_{j}\right|-\frac{1}{T}\left|x_{j}-\text{NH}{\left(x\right)}_{j}\right|, \end{array}$$

where *w*_*j*_ represents the weight of the *j*th feature and *T* represents the maximum number of iterations. ∣*x*_*j*_ − *y*_*j*_∣ is used to calculate the difference between the *j*th dimensional eigenvalues of two instances, that is, the absolute value vector of the feature difference vector.

A variant that considers *k* neighbors has been developed from the nearest neighbor Relief, whose weight value update formula is

(11) wj=wj+∑z∈KNNx,l,l∈cxj−zj/T−∑z∈KNNx,cxj−zj/T,

where KNN(*x*; *c*) is the set of *k* nearest neighbors of *x* in *X*_*c*_ by Euclidean distance. Process is shown in Algorithm 2.

### 3.2. Selection and Crossover Operator

The selection operator is to inherit the individuals with high fitness in the current population to the next generation according to selection probability. Generally, individuals with high fitness will have more chances to inherit to the next generation. This paper uses the roulette model to select individuals. The calculation formula is as follows:

(12) $$\begin{array}{c} p\left(x_{i}\right)=\frac{f\left(x_{i}\right)}{\sum_{j=1}^{n}f\left(x_{j}\right)}, \end{array}$$

(13) $$\begin{array}{c} q_{i}=\overset{i}{\underset{j=1}{\sum }}p\left(x_{j}\right), \end{array}$$

where *p*(*x*_*i*_) is the selection probability, *q*_*i*_ is the cumulative probability, *f*(*x*_*i*_) is the individual *x*_*i*_ fitness function value, and *n* is the number of the group. Select operator process is in Algorithm 3.

Crossover is to cross the selected a pair of individuals according to probability, such as single-point crossover or multipoint crossover. In this paper, the single-point crossover is adopted, that is, the random number is generated within the range of individual coding bits as the crossover point, and then, the coding exchange of the two bodies from this point to the end is carried out, so that the crossover process can be completed.

### 3.3. Weight-Based Elite Hybrid Binary Cuckoo Search (EHBCS) Algorithm

In the CS algorithm, the Lévy flight is used to explore the search space using a straight flight path with a sudden 90-degree turn, and Figure 1 simulates Lévy's flight path. In addition, the CS algorithm is highly dependent on random walk search, which can be easily moved from one area to another without carefully exploring each nest. Therefore, the CS algorithm has weak local search ability and low optimization accuracy [31]. In order to cover the mentioned weakness of the CS, elite strategy and genetic algorithm operators are embedded into the cuckoo algorithm, such as selection and crossover operators, so that the well-positioned nests can be inherited to the next generation. The so-called elitist strategy is to preserve the nest in a good location so as not to miss the optimal nest during the algorithm iterations by Lévy flight. According to certain rules, the selection operator is to inherit the individuals with high fitness in the current population to the next generation. Generally, individuals with high fitness will have more chances to inherit to the next generation. The crossover operator usually inputs two individuals as candidate solutions with a certain probability and generates neighborhood solutions by exchanging part of the chromosomes of two individuals.

The CS algorithm is suitable for continuous domain problems, and the feature selection is a binary discrete problem. This paper proposes an Elite Hybrid Binary Cuckoo Search (EHBCS) algorithm considering these facts. The EHBCS algorithm weights the features firstly according to the Relief algorithm mentioned in part III-A, so that the features with larger weights have greater opportunities to be selected. Then, in each iteration of the EHBCS algorithm, the optimal nest does not carry out Lévy flight or crossover to avoid damaging the optimal nest position. The nest generated by Lévy flight is operated by selection and crossover operators.

Since the existing BCS algorithm does not consider the influence brought by the Sig(step) function, the coefficient in the Sig(step) function is changed to the feature weight in this paper so that features with significant feature weight have a greater chance to be selected and the improved algorithm can finish the iterative process faster. The BCS mapping function is modified as follows:

When step ≥ 0

(14) $$\begin{array}{c} \text{sig}\left(\text{step}\right)=\frac{1}{1+e^{-\gamma \text{step}}},\gamma =w_{j}, \end{array}$$

(15) $$\begin{array}{c} x_{ij}^{t}=\left\{\begin{array}{c} \begin{array}{cc} 1 & \mathrm{rand}\left(\right)\leq \text{sig}\left(\text{step}\right)\\ 0 & \text{otherwise} \end{array}. \end{array}\right. \end{array}$$

When step < 0

(16) $$\begin{array}{c} \text{sig}\left(\text{step}\right)=1-\frac{1}{1+e^{-\gamma \text{step}}},\gamma =w_{j}, \end{array}$$

(17) $$\begin{array}{c} x_{ij}^{t}=\left\{\begin{array}{c} \begin{array}{cc} 1 & \mathrm{rand}\left(\right)\leq \text{sig}\left(\text{step}\right)\\ 0 & \text{otherwise} \end{array}. \end{array}\right. \end{array}$$

The function of sig(step) does not represent the probability of change, and it represents the probability of a certain change being 1. Let *γ* = −5, −3, 3, 5. The corresponding function graph is shown in Figure 2. It can be seen from the figure that the greater the parameter of the same abscissa, the greater the corresponding value. That is, the greater the feature weight, the greater the probability of being selected.

It should be emphasized that the weights calculated by the Relief algorithm may have negative weights, and the negative weight indicates that the distance of the similar neighbor samples is larger than that of the nonsimilar neighbor samples. Therefore, it is considered that this feature is unfavorable to classification, and the probability of selecting this feature in the corresponding feature selection is low.

Because the purpose of nest discovery and crossover operation is to make the population various, this paper adopts crossover operation instead of discovery operation. In the late iteration of the algorithm, the elite strategy proposed in this paper ensures the convergence. The elite selection and crossover operators as well as the pseudo-code of the algorithm presented in this paper are as follows: Algorithm 3 and Algorithm 4.

## 4. Experimental Methodology

### 4.1. Datasets

Eight datasets were extracted from the UCI Machine Learning Repository [33–35]. In order to make a more comprehensive comparison between the proposed algorithm and other algorithms, four low-dimensional feature datasets and four high-dimensional feature datasets are selected. Each dataset has two classes, and Table 1 provides the datasets' names, the total number of features, total number of cases, and classification accuracy before feature selection.

### 4.2. Performance Evaluation Measures

Generalization ability is the ability of a model to predict new data accurately after training on the training datasets. Cross-validation is a method to evaluate model generalization ability, which is widely used in data mining and machine learning [36]. In cross-validation, the dataset is usually divided into two parts: the training set, which is used to build a prediction model, and the other is test set, which is used to test the model's generalization ability. Cross-validation was performed, and the value of *k* was set to *k* = 5 for datasets with cases below 100 and to *k* = 10 for datasets with cases above 100. The evaluation indicators used include Accuracy, Sensitivity, Precision, and F-measure [37].

(18) $$\begin{array}{c} \text{accuracy}=\frac{\text{TP}+\text{TN}}{\text{TP}+\text{TN}+\text{FP}+\text{FN}}, \end{array}$$

(19) $$\begin{array}{c} \text{sensitivity}=\text{recall}=\frac{\text{TP}}{\text{TP}+\text{FN}}, \end{array}$$

(20) $$\begin{array}{c} \text{specificity}=\frac{\text{TN}}{\text{FP}+\text{TN}}, \end{array}$$

(21) $$\begin{array}{c} \text{precision}=\frac{\text{TP}}{\text{TP}+\text{FP}}, \end{array}$$

(22) $$\begin{array}{c} F-\text{measure}=\frac{2*\left(\text{precision}*\text{recall}\right)}{\text{precision}+\text{recall}}, \end{array}$$

whereTPis the total number of positive cases and correctly identified as positive,TNis the total number of negative cases and correctly identified as negative,FPis the total number of negative cases and wrongly identified positive cases, andFNis the total number of positive cases and wrongly identified negative cases.

For the overall classification performance of each algorithm, we calculate the average value of all tests as follows:

(23) $$\begin{array}{c} \text{acc}=\frac{1}{k}\overset{k}{\underset{i=1}{\sum }}\text{accurac}{\text{y}}_{i}, \end{array}$$

(24) $$\begin{array}{c} \text{SE}=\frac{1}{k}\overset{k}{\underset{i=1}{\sum }}\text{sensitivit}{\text{y}}_{i}, \end{array}$$

(25) $$\begin{array}{c} \text{SP}=\frac{1}{k}\overset{k}{\underset{i=1}{\sum }}\text{specificit}{\text{y}}_{i}, \end{array}$$

(26) $$\begin{array}{c} \text{Pre}=\frac{1}{k}\overset{k}{\underset{i=1}{\sum }}\text{precisio}{\text{n}}_{i}, \end{array}$$

(27) $$\begin{array}{c} F1=\frac{1}{k}\overset{k}{\underset{i=1}{\sum }}F-\text{measur}{\text{e}}_{i}, \end{array}$$

where *k* is the total number folds.

### 4.3. Evaluating Classification Performance

The support vector machine (SVM) classifier was adopted to evaluate the accuracy of feature subset classification. SVM is a supervised machine learning algorithm introduced by Boser et al. [38], in which data is mapped as the points in an *n*-dimensional feature space (*n* = number of features). The final output of SVM is an optimal hyperplane that classifies new cases.

SVM highly depends on kernel functions, so the experiments with different kernel functions are fundamental. The kernel function is a similarity function, which determines the similarity between any two inputs by calculating the distance between them. It is not difficult to determine the kernel function. Any function that satisfies the Mercer theorem can be used as a kernel function. There are various types of kernel functions such as linear kernel function, polynomial kernel function, radial basis kernel function, Sigmoid kernel function, and composite kernel function. Selecting the appropriate kernel function is relevant to the datasets and the problems. Therefore, it is often selected experimentally. Based on experiments, suitable kernel functions are selected to evaluate the datasets. The selected kernel functions are presented in Table 2.

### 4.4. Fitness Function

The main objective of the feature selection task is to find a subset of features from the dataset so that the learning algorithm can use these selected features to achieve as high accuracy as possible.

In the classification problems, two feature subsets with different numbers likely have the same classification accuracy for the same dataset. Therefore, in the case of the same classification accuracy, if the metaheuristic algorithm finds the subset with more features earlier, the subset with fewer features will be ignored. In this paper, a new evaluation method is proposed as the fitness function to overcome this constraint, which considers the classification accuracy and takes the rate of feature reduction as an adjusting term.

Let *d* be the total number of features contained in the datasets, *s* be the number of features selected by metaheuristic optimization algorithms, *β* be the weight of rate of feature reduction, and 1-*β* be the weight of average accuracy. The value of the adaptation fitness function can be calculated as shown in (28). We set *β*=0.2.

(28) $$\begin{array}{c} f=\beta \cdot \frac{d-s}{d}+\left(1-\beta \right)\cdot \text{acc}. \end{array}$$

### 4.5. Parameter Setting

The performance of the proposed EHBCS is compared against the Binary Genetic Algorithm (BGA) and Binary Particle Swarm Optimization (BPSO) algorithms.  Table 3 lists the parameter values for each algorithm. The population size of all optimization algorithms is set to 30, and each algorithm was run 5 times to perform the feature selection task. All runs are executed in Matlab 2017, running on a Windows 10 operating system on a Huawei MagicBook with Intel(R) Core(TM) i5-8250U 1.6GHz with 8Gb of RAM.

### 4.6. Analysis of Computational Complexity

The EHBCS algorithm uses the Relief algorithm and the binary conversion of Lévy flight as well as the selection and crossover process. For the Relief algorithm, assuming that the number of runs is *M*, the number of iterations is *m*, the number of cases is *N*, and the individual dimension is *d*; the complexity of the algorithm is *O*(*m* × *N* × *d* × *M*). For Lévy flight and binary conversion, assuming that the number of individuals is *n*, the individual dimension is *d*, and the number of iterations is *t*; the computational complexity is *O*(*n*^2^ × *d* × *t*). For selection and crossover, assuming the number of individuals is *n*, the computational complexity is *O*(*n*^2^ × *t* × *d*). Therefore, the computational complexity is *O*(*m* × *N* × *d* × *M* + *n*^2^ × *t* × *d*) for EHBCS algorithm.

## 5. Experimental Results

Figures 3 and 4 provide the performance of all optimization algorithms for feature selection using the medical datasets described in Section 4.1. They contain the following information:

*Accuracy*: classification accuracy for each datasets

*All*: classification accuracy before feature selection for each dataset

*SR*: size reduction percentage is used to evaluate the percentage of removed features compared to all available features

Tables 4 and 5 provide the performance of all optimization algorithms for feature selection using binary label datasets described in Section 4.1. Each table column contains the following information:

*Fitness*: acc is accuracy as defined in Section 4.2 Function (23), and *f* is the proposed Function (28) as defined in Section 4.4

*Algorithm*: it provides the abbreviations of the algorithms, Elite Hybrid Binary Cuckoo Search (EHBCS), Binary Genetic Algorithm (BGA), and Binary Particle Swarm Optimization (BPSO)

*Avgacc, Max, Min*: average accuracy, maximum accuracy, minimum accuracy of an algorithm during the 5 runs

*Std*: standard deviation of classification accuracy

*AvgN*: average number of features returned by the algorithm during the 5 runs

*SE, SP, Pre, F1*: average sensitivity, specificity, precision, *F*-measure of an algorithm during the 5 runs

*Dataset*: the dataset used for experimentation as described in Table 1

*Avg*: average of all corresponding data obtained by the three algorithms

The experimental results show that the average feature subsets are smaller for all datasets, and the average classification accuracy is improved to different degrees. Compared with the original datasets, the number of the average feature subsets after feature selection by the optimization algorithms was reduced by about 18.395%-89.667%, and the average classification accuracy was improved by about 3.3%-34.6%. For the Breast Cancer Wisconsin (diagnostic) dataset, the maximum average classification accuracy improvement was achieved at 34.6%. All these imply that the feature selection methods based on metaheuristic optimization algorithms can effectively eliminate redundant features and significantly improve the classification accuracy especially for some datasets.

For low-dimensional datasets, such as Cervical Cancer Behavior Risk, Breast Cancer Wisconsin (diagnostic), Breast Cancer Wisconsin (prognosis), and Sonar, the EHBCS algorithm can effectively reduce features to obtain a smaller subset of target features. It can get minimum standard deviation in three algorithms, which shows the EHBCS algorithm is the most stable of three. But it is the second of the three optimization algorithms in terms of classification accuracy, SE, SP, Pre, and F1. Compared with the data corresponding to Avg, the EHBCS algorithm has minimum standard deviation, higher classification accuracy, SE, SP, Pre, and F1 in entirety. Compared with the original dataset classification, the number of subset features after feature selection by the EHBCS algorithm is reduced by 58.182%-80%, and the classification accuracy is improved by 5%-33.9%. The results show that the EHBCS algorithm can efficiently diminish the number of features to ensure accuracy, but it did not perform well in low-dimensional datasets.

For high-dimensional datasets, such as Colon Tumor, Medulloblastomas, Central Nervous System and Relation Leukemia, the average classification accuracy, standard deviation, SE, SP, Pre, and F1 obtained by the EHBCS algorithm were superior to BGA and BPSO on the whole. Compared with the data corresponding to Avg, the average classification accuracy of the EHBCS algorithm is improved by 1%-10.6%, and the EHBCS gets lower standard deviation. But it needs to be explained that the standard deviation of the EHBCS algorithm is greater than the data corresponding to Avg when adopting fitness acc (Function (23)) for dataset Medulloblastomas and Central Nervous System. In addition to these, SE, SP, Pre, and F1 are optimal overall. Compared with the original dataset classification, the number of subset features after feature selection by the EHBCS algorithm is reduced by 43.772%-53.498%, and the classification accuracy is improved by 4.5%-22.8%. The results show that the feature selection method based on EHBCS has higher classification accuracy, SE, SP, Pre, F1, and smaller standard deviation. EHBCS algorithm is more suitable for the feature selection of high-dimensional datasets.

It should be emphasized that the purpose of feature selection is to reduce irrelevant or weakly correlated features as much as possible on the premise of ensuring classification accuracy. However, the number of feature subsets cannot be reduced indefinitely. Too few feature subsets may lead to the loss of important features, thus affecting the classification accuracy of the datasets. Therefore, it is necessary to balance the relationship between classification accuracy and the number of feature subsets. In practical applications, evaluation function models should be set scientifically and reasonably to ensure the classification performance of feature subsets.

## 6. Conclusion

This paper proposes an Elite Hybrid Binary Cuckoo Search Algorithm that adopts feature weighting and elite strategy. The proposed EHBCS algorithm aims to optimize the feature selection task on binary label datasets. The experimental results show that EHBCS achieves a better classification performance. Besides, all statistical metrics (standard deviation (Std), sensitivity (SE), specificity (SP), precision (Pre), and *F*-measure (*F*1)) reveal markedly the EHBCS is superior to BGA and BPSO. However, the algorithm still has shortcomings, such as increased computational complexity.

Future work requires further modification of the proposed algorithm to make it suitable for feature selection of multiclass datasets and to evaluate the results using different datasets and classification models.

## Figures and Tables

**Figure 1:** Lévy flight path.

**Figure 2:** Parameter comparison.

**Figure 3:** Accuracy and size reduction (%) with function *f*.

**Figure 4:** Accuracy and size reduction (%) with function acc.

**Algorithm 1:** Classical version of CS adapted from [15].

**Algorithm 2:** Relief algorithm.

**Algorithm 3:** Elite selection and crossover operators.

**Algorithm 4:** EHBCS algorithm.

**Table 1:** Datasets.

Datasets	Features	Cases	Accuracy
Cervical Cancer Behavior Risk	19	72	0.865
Breast Cancer Wisconsin (diagnostic)	30	569	0.627
Breast Cancer Wisconsin (prognosis)	33	198	0.763
Sonar	60	208	0.702
Colon Tumor	2000	62	0.853
Medulloblastomas	5893	34	0.648
Central Nervous System	7129	60	0.600
Relation Leukemia	7129	72	0.919

**Table 2:** Selected kernel functions.

Dataset	Kernel function
Cervical Cancer Behavior Risk	Radial basis function
Breast Cancer Wisconsin (diagnostic)	Radial basis function
Breast Cancer Wisconsin (prognosis)	Radial basis function
Sonar	Radial basis function
Colon Tumor	Linear function
Medulloblastomas	Linear function
Central Nervous System	Linear function
Relation Leukemia	Linear function

**Table 3:** Parameter setting.

Algorithms	Parameters
EHBCS	*α* = 1, *p*_*c*_ = 0.5, *p*_*r*_ = 0.3, *k* = 3
BGA	*p*_*c*_ = 0.8, *p*_*m*_ = 0.1
BPSO	*c*_1_ = 1, *c*_2_ = 2, *ω* = 0.9

**Table 4:** Experimental results.

Fitness	Algorithm	Avgacc	Max	Min	Std	AvgN	SE	SP	Pre	F1	Dataset
*f*	EHBCS	0.937	0.920	0.948	0.011	6.000	0.840	0.966	0.895	0.854	Cervical Cancer Behavior Risk
	BGA	0.954	0.975	0.934	0.015	5.000	0.917	0.952	0.906	0.893	
	BPSO	0.925	0.946	0.896	0.014	4.400	0.700	0.978	0.967	0.775	
	Avg	0.937	0.947	0.926	0.013	5.133	0.819	0.965	0.908	0.841	
acc	EHBCS	0.924	0.932	0.906	0.011	6.600	0.785	0.960	0.821	0.793	
	BGA	0.960	0.973	0.945	0.009	5.600	0.883	0.981	0.943	0.896	
	BPSO	0.920	0.948	0.896	0.017	5.300	0.753	0.917	0.800	0.754	
	Avg	0.935	0.951	0.916	0.012	5.833	0.807	0.953	0.854	0.814	
*f*	EHBCS	0.957	0.961	0.953	0.003	6.000	0.947	0.960	0.936	0.940	Breast Cancer Wisconsin (diagnostic)
	BGA	0.968	0.975	0.960	0.005	3.100	0.970	0.955	0.926	0.947	
	BPSO	0.962	0.972	0.954	0.006	5.600	0.954	0.941	0.907	0.930	
	Avg	0.962	0.969	0.956	0.005	4.900	0.953	0.952	0.923	0.939	
acc	EHBCS	0.966	0.968	0.963	0.001	8.200	0.957	0.969	0.950	0.952	
	BGA	0.973	0.977	0.968	0.003	7.900	0.954	0.959	0.940	0.952	
	BPSO	0.911	0.935	0.879	0.020	16.400	0.957	0.961	0.937	0.946	
	Avg	0.950	0.960	0.937	0.008	10.833	0.956	0.963	0.942	0.948	
*f*	EHBCS	0.787	0.793	0.778	0.007	10.200	0.294	0.926	0.604	0.371	Breast Cancer Wisconsin (prognosis)
	BGA	0.831	0.848	0.808	0.010	9.500	0.200	0.958	0.593	0.277	
	BPSO	0.814	0.825	0.793	0.014	10.800	0.216	0.936	0.583	0.286	
	Avg	0.811	0.822	0.793	0.010	10.167	0.236	0.940	0.593	0.311	
acc	EHBCS	0.797	0.803	0.793	0.005	13.800	0.220	0.974	0.750	0.322	
	BGA	0.822	0.863	0.788	0.020	13.500	0.210	0.981	0.735	0.302	
	BPSO	0.806	0.829	0.793	0.010	15.200	0.191	0.968	0.733	0.289	
	Avg	0.808	0.832	0.791	0.012	14.167	0.207	0.974	0.739	0.304	
*f*	EHBCS	0.755	0.778	0.735	0.017	15.200	0.947	0.960	0.936	0.940	Sonar
	BGA	0.816	0.880	0.778	0.036	11.000	0.970	0.955	0.926	0.947	
	BPSO	0.637	0.663	0.610	0.018	25.200	0.954	0.941	0.907	0.930	
	Avg	0.736	0.774	0.708	0.024	17.133	0.952	0.502	0.704	0.789	
acc	EHBCS	0.752	0.773	0.730	0.014	16.600	0.957	0.969	0.950	0.952	
	BGA	0.800	0.865	0.760	0.035	13.400	0.954	0.959	0.940	0.945	
	BPSO	0.631	0.644	0.620	0.009	27.600	0.967	0.961	0.937	0.946	
	Avg	0.728	0.761	0.703	0.019	19.200	0.974	0.451	0.684	0.788	

**Table 5:** Experimental results.

Fitness	Algorithm	Avgacc	Max	Min	Std	AvgN	SE	SP	Pre	F1	Dataset
*f*	EHBCS	0.899	0.901	0.886	0.006	931.833	0.927	0.860	0.938	0.922	Colon Tumor
	BGA	0.893	0.901	0.885	0.008	905.000	0.927	0.860	0.925	0.922	
	BPSO	0.877	0.886	0.868	0.008	984.300	0.927	0.753	0.888	0.901	
	Avg	0.889	0.896	0.879	0.007	933.744	0.927	0.824	0.917	0.915	
acc	EHBCS	0.898	0.903	0.886	0.006	1103.800	0.927	0.860	0.925	0.922	
	BGA	0.893	0.903	0.886	0.011	1033.000	0.927	0.860	0.905	0.901	
	BPSO	0.884	0.901	0.869	0.009	1632.100	0.927	0.793	0.910	0.913	
	Avg	0.892	0.902	0.881	0.007	1256.300	0.927	0.838	0.913	0.912	
*f*	EHBCS	0.876	0.876	0.876	0	2776.200	0.920	0.600	0.931	0.916	Medulloblastomas
	BGA	0.807	0.842	0.783	0.022	2798.600	0.920	0.600	0.931	0.917	
	BPSO	0.758	0.795	0.733	0.019	2927.800	0.910	0.600	0.921	0.912	
	Avg	0.814	0.838	0.797	0.014	2834.200	0.917	0.600	0.928	0.915	
acc	EHBCS	0.862	0.876	0.848	0.014	2899.800	0.910	0.550	0.915	0.907	
	BGA	0.798	0.817	0.783	0.015	2960.100	0.900	0.600	0.931	0.941	
	BPSO	0.764	0.767	0.762	0.002	3323.750	0.900	0.600	0.898	0.894	
	Avg	0.808	0.820	0.798	0.010	3061.217	0.903	0.583	0.915	0.914	
*f*	EHBCS	0.740	0.750	0.733	0.008	3315.100	0.436	0.894	0.767	0.525	Central Nervous System
	BGA	0.672	0.700	0.650	0.017	3425.300	0.360	0.794	0.430	0.380	
	BPSO	0.640	0.683	0.617	0.024	3569.100	0.360	0.737	0.396	0.360	
	Avg	0.684	0.711	0.667	0.016	3436.500	0.385	0.808	0.532	0.422	
acc	EHBCS	0.740	0.767	0.717	0.017	3693.600	0.500	0.894	0.787	0.572	
	BGA	0.670	0.717	0.633	0.023	3561.400	0.360	0.786	0.706	0.369	
	BPSO	0.643	0.650	0.633	0.008	4844.200	0.320	0.737	0.377	0.332	
	Avg	0.684	0.711	0.661	0.016	4033.067	0.393	0.806	0.623	0.425	
*f*	EHBCS	0.971	0.973	0.960	0.005	3482.000	1	0.930	0.953	0.975	Relation Leukemia
	BGA	0.970	0.973	0.960	0.006	3401.400	1	0.885	0.922	0.955	
	BPSO	0.952	0.960	0.947	0.007	3563.100	1	0.910	0.937	0.965	
	Avg	0.962	0.969	0.956	0.006	3482.167	1	0.908	0.937	0.965	
acc	EHBCS	0.973	0.987	0.960	0.006	4008.500	1	0.926	0.951	0.973	
	BGA	0.971	0.973	0.960	0.005	3573.100	1	0.910	0.937	0.965	
	BPSO	0.955	0.960	0.947	0.007	5661.200	1	0.910	0.937	0.965	
	Avg	0.967	0.973	0.956	0.006	4414.267	1	0.915	0.942	0.968	

## Data Availability

The data are available at the dataset site: http://archive.ics.uci.edu/mlhttp://portals.broadinstitute.org/cgi-bin/cancer/datasets.cgihttp://csse.szu.edu.cn/staff/zhuzx/Datasets.html.

## References

[1] Li Z. Q., Du J. Q., Nie B., Xiong W., Hung C., Li H. (2019). Summary of feature selection methods. *Computer Engineering and Application*.

[2] Liu H., Setiono R. A probabilistic approachto feature selection: a filter solution.

[3] Liu H., Zhou M. C., Liu Q. (2019). An embedded feature selection method for imbalanced data classification. *IEEE/CAA Journal of Automatica Sinica*.

[4] Kohavi R., John G. H. (1997). Wrappers for feature subset selection. *Artificial Intelligence Journal*.

[5] Chuang L. Y., Tsai S. W., Yang C. H. (2011). Improved binary particle swarm optimization using catfish effect for feature selection. *Expert Systems with Applications*.

[6] Bangyal W. H., Ahmad J., Shafi I., Abbas Q. (2012). A forward only counter propagation network-based approach for contraceptive method choice classification task. *Journal of Experimental and Theoretical Artificial Intelligence*.

[7] Zhao Q. F., Zhang Y. L. (2020). Ensemble method of feature selection and reverse construction of gene logical network based on information entropy. *International Journal of Pattern Recognition and Artificial Intelligence*.

[8] Liu J. X., Zhang Y. L. (2020). An attribute-weighted Bayes classifier based on asymmetric correlation coefficient. *International Journal of Pattern Recognition and Artificial Intelligence*.

[9] Zhang Y. L., Feng T., Wang S. (2020). A novel XGBoost method to identify cancer tissue-of-origin based on copy number variations. *Frontiers in genetics*.

[10] Rodrigues D., Pereira L. A. M., Almeida T. N. S. BCS: a binary cuckoo search algorithm for feature selection.

[11] Holland J. H. (1992). *Adaptation in Natural and Artificial Systems: An Introductory Analysis with Applications to Biology, Control and Artificial Intelligence*.

[12] Kennedy J., Eberhart R. Particle swarm optimization.

[13] Bangyal W. H., Ahmad J., Rauf H. T. (2019). Optimization of neural network using improved bat algorithm for data classification. *Journal of Medical Imaging and Health Informatics*.

[14] Junaid M., Bangyal W. H., Ahmad J. A novel Bat Algorithm using sobol sequence for the initialization of population.

[15] Yang X. S., Deb S. Cuckoo search via Levy flights.

[16] Liu Y., Xueming L., Zhang W., Peng J., Liao X., Zhongfu W. U. (2003). Feature subset selection based on genetic algorithm. *Computer Engineering*.

[17] Siedlecki W., Sklansky J. (1989). A note on genetic algorithms for large-scale feature selection. *Pattern Recognition Letters*.

[18] Kennedy J., Eberhart R. C. A discrete binary version of the particle swarm algorithm.

[19] Firpi H. A., Goodman E. (2004). Swarmed feature selection. *International Symposium on Information Theory*.

[20] Yang X. S., Deb S. (2014). Cuckoo search: recent advances and applications. *Neural Computing and Applications*.

[21] Civicioglu P., Besdok E. (2013). A conceptual comparison of the cuckoo-search, particle swarm optimization, differential evolution and artificial bee colony algorithms. *Artificial Intelligence Review*.

[22] Valian E., Mohanna S., Tavakoli S. (2011). Improved cuckoo search algorithm for feed forward neural network training. *International Journal of Artificial Intelligence & Applications*.

[23] Vazquez R. A. Training spiking neural models using cuckoo search algorithm.

[24] Pauline O. (2014). Adaptive cuckoo search algorithm for unconstrained optimization. *The Scientific World Journal*.

[25] FENG D., RUAN Q., du L. (2013). Binary cuckoo search algorithm. *Journal of Computer Applications*.

[26] Gherboudj A., Layeb A., Chikhi S. (2012). Solving 0-1 knapsack problems by a discrete binary version of cuckoo search algorithm. *International Journal of Bio Inspired Computation*.

[27] Pereira L. A. M., Rodrigues D., Almeida T. N. S. (2014). A Binary Cuckoo Search and Its Application for Feature Selection. *Cuckoo Search and Firefly Algorithm*.

[28] Bhattacharjee K. K., Sarmah S. P. A binary cuckoo search algorithm for knapsack problems.

[29] Sudha M. N., Selvarajan S. (2016). Feature selection based on enhanced cuckoo search for breast cancer classification in mammogram image. *Circuits and Systems*.

[30] Aziz M. A. E., Hassanien A. E. (2018). Modified cuckoo search algorithm with rough sets for feature selection. *Neural Computing and Applications*.

[31] Salesi S., Cosma G. A novel extended binary cuckoo search algorithm for feature selection.

[32] Kira K., Rendell L. A. A practical approach to feature selection.

[33] Lichman M. (2020). UCI machine learning repository. http://archive.ics.uci.edu/ml/.

[34] Medulloblastomas (2020). Cancer program datasets. http://portals.broadinstitute.org/cgi-bin/cancer/datasets.cgi/.

[35] High-dimentional datasets Microarray Datasets in Weka ARFF format. http://csse.szu.edu.cn/staff/zhuzx/Datasets.html/.

[36] Yadav S., Shukla S. Analysis of k-fold cross-validation over hold-out validation on colossal datasets for quality classification.

[37] Magna G., Casti P., Jayaraman S. V. (2016). Identification of mammography anomalies for breast cancer detection by an ensemble of classification models based on artificial immune system. *Knowledge Based Systems*.

[38] Boser B. E., Guyon I. M., Vapnik V. N. A training algorithm for optimal margin classifiers.

